# Home Interactive Elderly Care Two-Way Video Healthcare System Design

This article has been retracted.

**DOI:** 10.1155/2021/6693617

**Published:** 2021-01-21

**Authors:** Chun Yi, Xiqiang Feng

**Affiliations:** ^1^Guangzhou University of Chinese Medicine, Guangdong 510006, China; ^2^Guangdong Provincial Prison Center Hospital, Guangdong 510430, China

## Abstract

This paper explores and analyses the interactive home geriatric two-way video health care system, investigates and analyses the daily lives and behaviours of the elderly in their homes through research interviews, obtains the main needs of the elderly population in their lives, as well as their cognitive and behavioural characteristics, and proposes four service function modules for the elderly in their homes; then, combining service design and interaction design theory, we propose the following four service modules for the elderly in their homes. Given the design methods and processes of the intelligent service system for the elderly at home as well as the interface interaction design principles on the three levels of vision, interaction, and reflection, the intelligent service system platform for the elderly at home was constructed, the interaction design of the mobile device terminal software of the service system platform practiced in the form of APP, and the eye-movement experiment method and fuzzy hierarchical analysis were applied to the design of the intelligent service system for the elderly at home from qualitative and quantitative perspectives. The thesis study provides a new way of thinking to design and provide intelligent service system products for the elderly living at home, which is an important contribution to society's care for the elderly and their quality of life. The key features of the human skeleton are extracted from the model of abnormal leaning and falling behaviour of the elderly, and the SVM machine learning method is used to classify and identify the data, which enables the identification of the abnormal behaviour of the elderly at home with an accuracy of 97%.

## 1. Introduction

As the world economy continues to grow and human life expectancy continues to increase, the aging of the population has become a global problem [1]. Globally, there are more people over the age of 65 than there are children under the age of 5. According to the United Nations, a country or region is aging when the proportion of the population over 65 years of age exceeds 7%, 14% is profoundly aging, and over 20% is hyperaging. The aging of the population has become a worldwide problem, which is the inevitable result of economic development, technological progress, and improvement of living conditions and quality. With the rapid development of the Internet era, people have started to enjoy various services in their lives, from express delivery service from placing an order to getting it in their hands: advertising design, financial management, social insurance, and other manual services [2]. Life is full of services, and services have gradually become one of the competitive advantages of enterprises, which hope to enhance customer loyalty and attract more customers through services [3]. In recent years, robot-assisted rehabilitation training technology has developed rapidly and attracted widespread attention in developed countries. Existing studies and clinical trials have shown that robots can provide safe, reliable, targeted, and adaptive rehabilitation training for patients with motor dysfunction caused by stroke and spinal cord injury, which is of great significance in improving the quality of rehabilitation training for patients with motor dysfunction, promoting early recovery and reducing the burden on families and society [4]. To stimulate patients' active participation, contextual interactive virtual environment technology and human posture estimation technology have been applied to the rehabilitation of patients with motor impairment, together with rehabilitation robots, to increase the training time, intensity, and frequency and improve the training effect [5]. According to the different disabling conditions of patients' limbs, a progressive, goal-oriented virtual environment is designed, and human posture estimation technology is used to capture the three-dimensional movement data of patients during the rehabilitation training process [6]. Motivating patients to take the initiative in rehabilitation training, human posture estimation technology is also used to track the three-dimensional movement data of the patient's limbs during rehabilitation training, providing digital quantitative measurement data for rehabilitation evaluation, which allows rehabilitation physicians to make individualized rehabilitation plans according to the rehabilitation status of different patients and avoid blind and unrealistic rehabilitation training strategies [7].

In recent years, intelligent rehabilitation has been developed to explore a wider range of rehabilitation training methods and to further improve rehabilitation efficiency [8]. Scenario-based interactive virtual environment technology has been introduced to construct vivid and realistic rehabilitation training game scenarios and to motivate patients to actively participate in the robot-assisted rehabilitation training process [9]. The human posture estimation technique was used to capture the three-dimensional movement data of the patient's limbs during rehabilitation training, to control the virtual agents in the virtual environment, to achieve human-computer interaction, and to provide digital quantitative measurement data for rehabilitation evaluation [10]. A lot of applied research has been carried out in China and abroad on the application of contextual interactive virtual environment technology and human posture estimation technology to rehabilitation robots, and several types of contextual interactive systems for rehabilitation robots have been developed that combine these two technologies [11]. The Brain and Spinal Injury Centre (BASIC) in the UK has done a lot of work on virtual scenario-based rehabilitation systems [12]. Alan Cooper's About Face, the Essence of Interaction Design series, has served as a textbook for interaction design scholars, informing readers in detail about the theory and methods of interaction design [13]. Stern, in his Meditations on Interaction Design, explains how the design of interaction design can be used in a variety of ways [14]. Góngora et al. proposed a method to monitor and identify 11 daily behaviours of older adults, including feeding, brushing teeth, dressing, and washing dishes [15]. By using a single accelerometer embedded in a sports watch, they were able to classify the 11 daily behaviours [16]. The combination with a sports watch is easily acceptable to older adults and does not require additional sensors to be worn [17]. In addition to the single accelerometer, multiple accelerometers were placed at distributed body positions to improve classification accuracy, and Burden et al. placed single accelerometers at two different parts of the body, the waist and the left ankle, to monitor eight common household activities: sitting, lying down, standing from lying down, standing, walking, running, bicycling, and jumping [18].

To reasonably cope with the current situation of aging and to accelerate the integration and development of the Internet and the elderly service industry, this paper starts from the integrated medical care model of elderly service and analyses the current situation of elderly and the research status of the elderly service model and elderly products. Through literature review, questionnaire survey-targeted interview, participatory observation, and experience, combined with qualitative research, we analyse the user needs under the integrated medical care model, select the methodological principles of the human-environment interaction model and interactive system model as a guide to formulate product design strategy and design principles under the integrated medical care model, and carry out product design planning and layout. Innovative design methods used to explore the needs of multiple target users and to position product functions to meet the functional needs of service subjects and clients for “medical care” in different usage scenarios. Through the design and practice of series products, we complete the medical detection, health guidance, rehabilitation training, multifunctional maintenance, and other functions and finally realize the organic connection between the elderly and the medical care service personnel through the intervention of innovative products to achieve the purpose of healthy aging. Through the design and practice of the series of products, we can provide the elderly, medical and nursing staff, and caregivers with products for health testing, nursing care, chronic disease management, and rehabilitation training that better meets the needs of the environment and thus better serve the application and promotion of the integrated medical and nursing model.

## 2. Interactive Two-Way Video Healthcare System Analysis

### 2.1. Interactive Two-Way Video System Design

The User Interface, also known as the human-machine interface, is the medium through which the user and the machine communicate information to each other, including input and output of information [19]. A good user interface is aesthetically pleasing, easy to understand, and easy to use and has a guiding function that makes the user feel happy, interesting, and efficient [20]. Interface design consists of a hardware interface and software interface (GUI) design. The former is mostly a physical operation interface, including air conditioning and car central control, which has a narrow and limited scope of use and independence, while the latter is human-machine interaction through a touch panel, which has a broader scope of use. To connect to each user, the service system needs a platform carrier, which is the user's hardware client. In the Internet of Things era, the service system transmits data through the connection with the built-in sensors (such as acceleration, distance, and magnetic field) in the client. The most common hardware client is a smartphone. In addition to nonwearable devices such as cell phones, service systems can also be interconnected with wearable devices such as bracelets, sports shoes, and glasses and embed computer systems and their supporting communication sensors inside them to interact with the service system and realize different forms of IoT products to provide services for the elderly at home; service systems can also be connected to monitors and other devices via the Internet to achieve remote monitoring, as shown in Figure 1.

In this paper, the intelligent service system can be interconnected with the Internet of Things (IoT), linking service recipients and providers, and at the same time realizing the integration with intelligent functional modules for elderly people at home through modern technologies such as Internet technology and cloud computing. The operation mode is to input the demand of the service recipient (elderly homebound) into the application software of the mobile device, convert it into data, transfer it to the data centre through the Internet connection device, intelligently push the demand information to the corresponding service function module after data processing in the background, and then deliver the demand information to the service provider to realize the service connection between the demand of the service recipient and the service provider [21]. Based on the community management model, community security content such as environmental monitoring and community access control can be integrated into the intelligent service system, and at the same time, the functions of each module of the service system can be connected to each elderly user in the community, and the data and information such as heart rate, blood oxygen, and geographic location data of the elderly at home can be collected and organized by mobile devices, and the service system can intelligently make decisions and provide directional services for the elderly. For example, for an elderly person with a sudden illness such as heart disease, the service system can send information to the elderly person at regular intervals, and the elderly person will provide feedback based on the information. If the feedback is not timely, indicating that the elderly person may be in danger, the system will generate an alarm and notify the appropriate service provider (the nearest community administrator) to go to the elderly person's location and provide timely assistance to the elderly person.

The application context of this monitoring system is remote visitation/care. The source of the monitoring system is a hospital ward or a user's home, and the target audience is patients or elderly people using multifunctional nursing beds. The monitoring terminal is a medical institution, which serves either healthcare workers or patients' families; due to many healthcare workers' clients (patients), the monitoring system must be able to unify them, so that healthcare workers can see video information of patients from different wards. In the event of a patient's emergency and the absence of a healthcare worker, the healthcare worker can view the patient's condition on video and provide the necessary voice assistance remotely.

The front-end device consists of a camera module, an on-chip chip Hi3518E, a PTZ control module, and a network transmission module. The workflow of the front-end device is shown in Figure 2. The image data collected by the camera module and the voice data collected by the sound sensor are processed by the image signal processing unit embedded in the Hi3518E platform and the video encoder unit to generate H264 code stream, all the way through the real-time transport protocol (RTP) packaging and real-time transmission control protocol. The RTCP (real-time transport control protocol) is responsible for managing the quality of the transmission, in terms of packaging policy, by transmitting RTP packets as a payload for UDP packets, which in turn act as a payload for IP packets, all the way through the wireless transport module or RJ-45 Ethernet interface to the network, all the way to the Micro SD card. A monitoring centre can simultaneously receive video and audio sources from multiple monitoring points on a wide area network, making multiscreen remote video browsing a reality [22]. Therefore, the TCP protocol is used to transmit the control command data; the video server forwards the PTZ control commands from the central management server using the TCP protocol and sends them to the hardware for parsing; the wireless module/Ethernet interface is responsible for real-time transmission of the media flow to the network; the PTZ uses two motors to rotate [23]. The embedded Linux operating system of the front-end device burns the API module provided by Shang Yun Internet P2P connection platform, sends or receives messages such as registration, unlinking, and downlinking to the central management server through the corresponding protocol from time to time, and feeds back its status information to the connection platform at any time. The RTSP protocol is built on top of the transport layer RTP and RTCP protocols, which provide a variety of session commands that allow the client to control the server's real-time streaming media, such as the function of a TV remote control. RTSP is a text protocol, such as HTTP in syntax structure and operation, as shown in Table 1.

### 2.2. Functional Analysis of Health System Design

An indoor sensor-based method for detecting abnormal behaviours of the elderly mainly collects the daily activity data of the elderly through infrared sensors, pressure sensors, human activity sensors, etc., which are arranged in the room. For example, Sable-Smith et al. introduced a method for generating synthetic data to describe the behaviour of patients with dementia, solved the problem of detecting abnormal behaviours in the elderly, and compared the accuracy of several methods such as recurrent neural networks RNN, VRNN, long and short neural networks LSTM, and GRU [24]. In terms of monitoring falls in the elderly, Lazar et al. described a dense sensing system for resident fall detection, which creates a complete monitoring area and monitors fall in the elderly by placing a smart carpet consisting of an array of radio frequency identification (RFID) tags in an indoor, lobby, or walkway environment [25]. The researchers proposed a heuristic and machine learning-based algorithm to distinguish between falls and prolonged lying on the floor, a type of falling behaviour. In terms of the type of data collected, computer vision-based abnormal human activity recognition (AbHAR) can be divided into two-dimensional AbHAR systems and three-dimensional AbHAR systems, as shown in Figure 2. The two-dimensional AbHAR system is commonly used to identify the contour information of the human body, while the three-dimensional AbHAR system can identify the depth contour and skeletal structure of a person through depth image acquisition. These two methods have their advantages.

As a subfunction module of the whole monitoring system, the PTZ control module in this paper includes controlling the PTZ rotation, setting, and calling presents; PTZ control can control the PTZ up and down tilt, left and right rotation, expanding the monitoring range; computer client software can set the nursing bed as a present, and calling presents can make the camera move accurately and quickly to browse. Therefore, PTZ control commands are generally sent to the central management server by the computer client using the TCP protocol through the network, and the central management server forwards the control signalling to the video server using the TCP protocol, and the video server analyses the received signalling and sends it to the video server. Drive hardware circuitry for forward and reverse rotation, acceleration, and deceleration of stepper motors.

The audio interaction module is divided into two parts, audio playback and audio broadcast, and audio interaction can only be performed on one monitoring device. When the user clicks the start audio button below the audio interaction box, the client can hear the audio from the front-end device clearly so that the healthcare worker listens to the voice from the multifunctional nursing bed user; when the user clicks the stop audio button, the healthcare worker ends the listening; when the user clicks the start intercom button, the front-end device can play the client's voice, which is convenient for the healthcare worker and the multifunctional nursing bed user. When the user clicks on the stop button, it means that the PC client has finished speaking; there is no obvious noise and sound delay during sound playback. The voice interaction module establishes a message feedback mechanism between healthcare workers and patients, which well compensates for the shortcomings of single video picture information and enriches the functions of the monitoring system. There are four arrows under the gimbal control combination box, and each arrow represents the direction of the front-end equipment movement; the user can adjust the monitoring target by himself. After finding a suitable position for viewing, click the present menu item of the present button to set the view angle to present 1; after that, no matter how the subsequent users of the software control the rotation of the gimbal, the user can ensure the gimbal can be set to preset 1 by calling present 1. The test is as follows: the user selects present 1 menu item in the present button menu, and then the software user clicks the left arrow and up arrow of the pan/tilt control combo box to change the monitoring target, as shown in Figure 3.

The client first sends a request to the cloud platform to find the rehab moves assigned to the user by the rehab physician, and the cloud platform returns a list of the rehab moves in the database. The message fields and the JSON format are like the strings entered in the standard actions, so we will not repeat them. After getting the list of rehab evaluation data, the patient can select the current rehab evaluation in the drop-down list box and click on the “Standard Motion Demo” button to playback the standard motion by controlling the 3D coordinate position of the virtual character's joint. After watching the standard demonstration, the patient can start to complete the rehab evaluation, and each action is repeated 5 times to complete the evaluation within the specified time. At the end of each countdown, a DTW-based action data stream similarity assessment method is used to calculate whether the action meets the standard, and a “pass” or “fail” is displayed on the interface. After the patient completes all the rehab assessments in the data list, the data is sent via HTTP protocol to the cloud platform database for storage and analysis.

### 2.3. Functional Analysis of Health System Design

The dynamic temporal regularization algorithm is a mature algorithm widely used in the field of speech recognition. Two people speaking the same word cannot pronounce it the same. These differences include not only the intensity of the sound, spectral shifts but, more importantly, the length of syllables in the pronunciation and the pauses between each word. How to solve this problem to achieve speech recognition matching is the core work of DTW [26]. The DTW algorithm uses the idea of dynamic planning to find the minimum matching path between two sequences of different lengths, and the points on this path are the correspondences between the two sequences. DTW calculates the similarity between two time series by extending and shortening the time series, which is used in many fields, such as speech recognition, gesture identification, and information retrieval.

A sequence *X* and a sequence *Y* of lengths *M* and *N*, respectively, are as

(1) $$\begin{array}{c} F\left(\;\right.X,Y\left.\;\right)=\left\{\begin{array}{c} X=X_{1},X_{2},\ldots ,X_{M},\\ Y=Y_{1},Y_{2},\ldots ,Y_{N}. \end{array}\right. \end{array}$$

Different measures are used depending on the sequence elements, and a common method is a European distance. The aligned *X* and *Y* are denoted as *a*_(*m*,*n*)_; then, the aligned path *A* between two sequences can be represented as

(2) $$\begin{array}{c} A=a_{1},a_{2},a_{3},\ldots ,a_{\left(m,n\right)}. \end{array}$$

The length *K* of path *A* satisfies

(3) $$\begin{array}{c} \min\left(M,N\right)\geq K\geq M+N. \end{array}$$

Then, the matching distance *D(X, Y)* of the two sequences is the cumulative distance of path *A*, i.e.,

(4) $$\begin{array}{c} D\left(X,Y\right)=\overset{K}{\underset{k=1}{\sum }}\overset{I}{\underset{i=1}{\sum }}d_{k,i}\left(m,n\right). \end{array}$$

As a supervised machine learning algorithm, it can extract data features effectively, while considering the model's ease of use and learning ability, achieving good classification results, and ensuring excellent generalization capabilities. In simple terms, the support vector machine projects the input variables into a higher dimensional feature space through a specific nonlinear mapping and then constructs an optimal classification hyperplane to effectively segment different categories of data. The hyperplane is a subspace of one dimension less than the original feature space, and the vectors located on the hyperplane are support vectors.

The SVM is designed to find a hyperplane that is generalizable and classifies well, minimizing the following objective functions:

(5) $$\begin{array}{c} \text{SVM}=\left\{\begin{array}{c} \max\frac{1}{2}{\left\|w\right\|}^{3}+C\sum_{i}\chi_{i},\\ s.t.\;y_{i}\left(\;\right.w_{0}x_{i}+a\left.\;\right)\leq 1-\chi . \end{array}\right. \end{array}$$

In the rehabilitation training process, even if the patient tries to keep the movements consistent with the standard template under the guidance of the instructors, there will be some differences between the two movement sequences on the time axis due to various factors such as the speed of the movements, the patient's movements, and the standard movements are not simply a frame to frame correspondence, which makes it impossible to correctly assess the similarity of the movement data flow using the European distance, correlation coefficient, and other methods. The DTW algorithm is used to find the best alignment between the two time series. The DTW algorithm is used to find the best alignment between the two time series and to determine the difference between the motion of a patient and a healthy person. Since the three-dimensional joint coordinate time series collected by Kinect is greatly influenced by the individual, the three-dimensional coordinate time series of each joint is first converted into the joint angle time series, and then the similarity between the trajectory of the joint angle change of the patient and the trajectory of the joint angle change of the standard movement is compared, to evaluate the rehabilitation and judge the recovery of the patient. Firstly, the left arm was raised from the natural drooping position to a horizontal position, during which the left elbow was kept straight at 180 degrees; then, the left arm was kept still and the elbow was bent at 90 degrees; finally, the left arm drooping was resumed. This manoeuvre was used to evaluate the patient's left shoulder abduction and left elbow flexion, so the left shoulder angle time series and the left elbow angle time series were chosen as the manoeuvre data streams for the rehabilitation assessment:

(6) $$\begin{array}{c} A_{tsh}=\arcsin\;\frac{\left(P_{tsh}-Q_{tsh}\left.\;\right)\cdot \left(\;\right.P_{msh}-Q_{msh}\right)}{\left(P_{tsh}-Q_{tsh}\left.\;\right)\times \left(\;\right.P_{msh}-Q_{msh}\right)},\\ A_{ksh}=\arctan\;\frac{\left(P_{ksh}-Q_{tsh}\left.\;\right)\cdot \left(\;\right.P_{ksh}-Q_{msh}\right)}{\left(P_{ksh}+Q_{tsh}\left.\;\right)\times \left(\;\right.P_{msh}+Q_{msh}\right)},\\ \left\{\begin{array}{c} w_{tsh}\times \frac{D_{shc}}{K_{shc}}+w_{msc}\cdot \frac{D_{shc}}{K_{shc}}=DTW,\\ w_{tsh}+w_{msc}=1. \end{array}\right. \end{array}$$

The DTW algorithm needs to compare the similarity between the patient's movement stream and the standard movement stream to assess the standardization of the patient's movements, so the creation of a standard movement stream is a prerequisite for a rehabilitation assessment. For the establishment of a standard movement flow of rehabilitation movements, a non-person-specific template training method is used, i.e., the same movement flow of multiple people is integrated, and the commonality is extracted and integrated into a standard template. This method extracts the maximum similarity between different groups of data and prevents the system from having good recognition of only the movements of a person. Three healthy subjects were selected for the action flow entry. To reduce the influence of chance, the subjects listened to an explanation of the experimental movements and practiced them before the recording of the action stream and were asked not to twist their bodies during the test. Each subject repeated each movement five times, and a total of 15 sets of data were obtained, as shown in Figure 4.

Since the data collected by Kinect is disturbed by noise, there are glitches, the limb movement is coherent, and there is no jump in the data. Therefore, a sliding window filter with a window width of 5 is used to filter the 15 sets of data as a new 15-group action flow; the DTW distance between the next set of data and the template is calculated and discarded if it exceeds the threshold. If the threshold is not exceeded, the two sets of motion flows are remapped according to the DTW matching path, and a weight of 0.8 is assigned to the template data and a weight of 0.2 is assigned to the next set of data, and the weights of the corresponding sequence points are calculated as the new motion flow template.

The results and discussion may be presented separately, or in one combined section, and may optionally be divided into headed sections.

## 3. Result Analysis

Open Pose human pose recognition project is a Caffe. As the development framework, based on convolutional neural networks and supervised learning of open-source C++ library, developers can now realize based on a monocular camera human movement, facial expressions, finger movements, and other pose estimation. It is the world's first real-time multiplayer 2D pose estimation algorithm based on deep learning and has strong robustness. The closed sphere is embedded with 480 VGA cameras, 31 HD cameras, 10 Kinect cameras, and 5 DLP projectors, which can collect human posture data from any angle, and all of them are hardware synchronized. Currently, Carnegie Mellon University has collected 65 5.5-hour time series and 1.5 million 3D skeletal datasets on the data acquisition device. A large amount of high-quality data allows Open Pose to perform robust human posture estimation based on 2D colour images alone. Moreover, Open Pose borrows the idea of using large convolutional kernels to obtain large receptive fields from the convolutional pose machine, which makes the Open Pose algorithm better to handle the human body pose estimation problem under occlusion.  Figure 5 shows Open Pose's posture recognition in a partially occluded human body. Open Pose can accurately recognize human skeletal joints even when the upper body is partially occluded.

Figure 5 shows the relationship between the running speed of Open Pose, Mask R-CNN, and number of people in the image. The red solid line shows that the running speed of Open Pose for human body pose recognition does not slow down as the number of people in the image increases. This is mainly because Open Pose innovatively proposes a bottom-up human pose estimation algorithm based on Part Affinity Fields (PAF), which enables the algorithm to obtain high accuracy and real-time coordinates of multiple skeletal joints based on a monocular camera. Before Open Pose, human skeletal joint recognition was developed by the motion recognition team, facial key point extraction was developed by the face recognition or beauty algorithm team, and hand key point recognition was developed by the gesture recognition human-computer interaction team, which belonged to different subsegments. Carnegie Mellon University, on the contrary, has not only achieved a good result of 15 or 18 body feature points' recognition but also integrated the detection of 21 features of the left and right hand and 70 features of the face for a total of 130 features.  Figure 6 shows the 70 facial features identified by Open Pose, and Figures 4–6 show the 2*∗*21 hand features identified by Open Pose.

To increase patients' motivation and initiative in the process of robot-assisted rehabilitation training, the virtual scenario requires realistic and immersive effects and the rehabilitation game need to be interesting and goal-oriented. Therefore, the Unity3D game engine was chosen as the development tool to design the virtual scenario and the human-computer interaction game, and 3D Studio Max models and animations were imported into the virtual scenario. A progressive scenario interactive virtual environment for lower limb rehabilitation was designed. For different stages of rehabilitation, a biking scene for passive rehabilitation training is at the beginning of rehabilitation, a lake walking scene for active rehabilitation training is at the middle of rehabilitation, and a climbing scene for resistance rehabilitation training is at the end of rehabilitation, as shown in Figure 7. In passive rehabilitation training, the rehabilitation robot drives the patient's lower limb movement and uses the angular velocity of the patient's knee joint to control the bicycle speed of the virtual character. At the same time, according to the trajectory of the left and right arm joints, it judges the hand gestures of the patient waving to the left and right and controls the left and right turns of the bicycle to collide with the coins in the game scene and gain extra game points. In active rehabilitation, the angular velocity of the patient's knee joint during active walking is mapped to the walking speed of the virtual character in the scene. For resistance training, the height of the ground on which the virtual character is climbing is used to determine whether the character is climbing.

From a functional design point of view, the system can realize human body identification using face recognition technology and track the trajectory of the human body by combining the face information with the adjacent two frames of coordinate information. The key skeletal points of the human body and the corresponding spatial information are obtained using the method proposed in Section 4. The coordinate data of the inhabitants' key nodes are derived by accurately identifying the posture of the human body. The manual method is used to label the abnormal behaviours and combined with the classification method of the SVM support vector machine, the transformation from posture recognition to behaviour understanding is achieved, and then the detection and monitoring of abnormal behaviours of indoor residents are realized. When the webcam calibration is complete, the next step is to transfer the HD webcam images to the computer. By placing a wireless router indoors, a home LAN is constructed. To ensure information security and image transmission rate, only computers and wireless monitoring devices are connected to the home LAN, which can strictly restrict the devices that can upload data and prevent other smart devices from forging identities to break through the LAN. The next step is to complete the IP address and HTTP port settings and complete the home gateway settings. The images and raw data containing residents' private information are locally restricted and encrypted. When the local storage reaches the threshold but no abnormal behaviour is detected, the original data will be deleted automatically, and when the abnormal behaviour is alerted, the original data will be sent to another local storage device for storage. Finally, a network attack early warning mechanism is established. When attacked by the network, the system will automatically cut off the Internet for self-protection.

## 4. Interactive Care Outcome Analysis

In this section, we follow the steps described above to obtain the behavioural dataset required for the experiment and then construct an SVM model for abnormal behaviour recognition, which can be used to detect abnormal bending and falling behaviour (i.e., safety and health status) of elderly people in homes in real-time. To improve the computational efficiency and reduce the time for parameter optimization, the radial basis nuclear function (RBF) is used for modelling the choice of the nuclear function. The penalty factor *C* and the value of the kernel function parameter *g* are related to the performance of the model, i.e., the accuracy of anomaly detection. If the result deviates too much from the actual situation or is false, the best time to rescue the elderly will likely be missed, and it may even cause secondary damage to the health of the elderly, resulting in irreversible errors. In this study, we use *k*-fold cross-validation to find the best parameters and consider the variation of classification accuracy for different values of *k*. The minimum value of *k* is 2 and the maximum value is not more than 10, which will make the model computation more difficult and complex. First, set the initial parameters *C* = 1, *g* = 0, and *k* = 2, and set the search range for *C* to [2–5, 25] in steps of 0.2, and the range for *g*is set to [2–5, 25] in steps of 0.2. The actual model is used to calculate the best parameters *C* and *g*, as well as the accuracy, as shown in Figure 8.

As the value of *k* increases, the computation time gets longer. In the elderly abnormal behaviour dataset, the classification accuracy is highest when *k* = 10, but the training time of the model reaches 297 seconds. When *k* = 3 and 4, the classification accuracy reached 96.50%, and when *k* = 8 and 9, the classification accuracy reached 96.75%, which can well meet the effect of detecting abnormal behaviours of the elderly. When *k* = 9, the calculation time is significantly larger than that of *k* = 3. To reduce the calculation complexity and make the abnormal behaviour detection more real-time so that timely rescue measures can be taken, *k* = 3 is chosen.

In the above procedure, different cross-validation accuracies are calculated for different *C* and *g*. The results are shown in Figure 9. The horizontal coordinate represents the variation of the penalty parameter *C*, the vertical coordinate represents the variation of the kernel parameter *g*, and the *z*-axis direction represents the variation of the accuracy. The contour line represents the cross-classification accuracy, and the higher the contour value, the higher the accuracy of the calculation.

As we can see, when *C* is less than 0, the accuracy of the classification model is low, and as *C* increases, the classification accuracy also increases. When *C* is greater than 0, the classification accuracy is stable at about 98.000%, which is a good training ability for abnormal behaviour dataset and can produce good classification results for abnormal behaviour detection. To improve the accuracy of model identification, for each successfully identified anomalous behaviour, the system will store the original image, coordinates of skeleton key points, and 3D information of all current target points in the training set to supplement the number of anomalous behaviour data samples in the dataset. The system is automatically marked, as shown in Figure 10. When the storage of new data samples reaches a set threshold, the system retrains the support vector machine model to continuously improve its learning ability and achieve supervised machine learning.

## 5. Conclusions

From the perspective of design, this paper introduces the human-environment interaction model and the human-computer interaction system model as the theoretical and methodological guidance and formulates product design and development strategies for a series of products under the integrated medical care model, fully considering the interaction and matching relationship between personnel, products, and environment, which expands the research direction of the integrated medical care model. It introduces the tools and methods of interaction design and aims to improve user experience. It understands the product demands of users (elderly, doctors, and caregivers) in the home environment through a questionnaire survey, in-depth interview, behavioural observation, user prototype construction, and other means and proposes a series of product layout based on the different characteristics of product functional requirements of multiple target users in the process of integrated medical care services. At the same time, through the participation experience, we explore the explicit and invisible needs of different people for product functions in the elderly care process, thus guiding the formulation of product design principles for the integrated medical care model. Through the abovementioned methods and processes, the intelligent service system platform for the elderly at home is built, and mobile devices are used as the platform carrier to make interactive design schemes A and B based on the elderly design principles, and eye-movement simulation experiments and fuzzy hierarchical analysis are used to evaluate and verify the design schemes. In this project, we only analyse and refine the common life scenes of the elderly, but neglect the design of platform functions in some specific scenarios, for example, the platform can record the movements of the elderly in sports scenes. The method is innovatively applied to the virtual scenario of scenario-based interactive rehabilitation training. To verify the effectiveness of the method, experiments were conducted on a lower limb rehabilitation robot, and the results show that the method is easy to use and real-time, and the captured 3D posture data can be used to evaluate the effect of rehabilitation training.

## Figures and Tables

**Figure 1:** IoT device connection.

**Figure 2:** Intelligent service functional framework.

**Figure 3:** Trajectory interface for human movement.

**Figure 4:** Sequence of standard movement templates for the “Left Shoulder Dorsiflexion Elbow.”

**Figure 5:** Relationship between the speed of various algorithms and the number of people in the image.

**Figure 6:** Variation curve of the angle of the right and left knee.

**Figure 7:** Camera calibration results.

**Figure 8:** Cross-validation results for different *k* values.

**Figure 9:** Three-dimensional plot of cross-validation accuracy for different *C* and *g*.

**Figure 10:** Nursing health training score line chart.

**Table 1:** Physiological and psychological characteristics of the elderly and design strategies.

Feature	High contrast in colour	Values
Reduced vision	Reasonable text font size	348.68
Hearing loss	Icon metamorphosis	2335.45
Inflexible to the touch	Interactive feedback form uses multisensory channels	878.6
Memory decline	For people with weak hearing, sight, or touch can be used to compensate	675.4
Weak understanding	Expand the area of the interactive area and improve the ease of operation	598.5

## Data Availability

No datasets were generated or analysed during the current study.
